# Health Index Monitoring of Sports Injury Rehabilitation Training Based on Wearable Sensors

**DOI:** 10.1155/2021/6302991

**Published:** 2021-09-29

**Authors:** Jiang Yi, Yuepei Zou

**Affiliations:** ^1^Institute of Education Beijing Sports University, Beijing, China; ^2^Institute of Physical Education, Hainan Normal University Haikou Hainan, Haikou, China; ^3^Department of Physical Education and Sport Sciences (Main Campus), Zhengzhou University, Zhengzhou, China; ^4^China Key Laboratory of Classification, Evaluation and Rehabilitation (Sport) of Intellectual and Developmental Disability, Zhengzhou, China

## Abstract

In order to design the perception system of the lower limb wearable rehabilitation robot, this study established the kinematics theoretical model of human lower limb and conducted the kinematics analysis of human body. By using the dynamic attitude analysis system, combined with the human body mark points, the position data of human body mark points in the process of standing up, sitting up, walking, stepping up, and squatting were collected. Combined with the movement mechanism of human lower limbs, the characteristics of human motion state transition are analyzed, and the perceptual algorithm for judging human motion intention is studied, so as to determine the wearer's current posture, standing intention while sitting, walking intention while standing, moving intention, and stopping intention during walking. The results show that the angle of the hip joint changes regularly between 0° and 37° and the angle of the knee joint changes regularly between 0° and 70°during the standing process, which is consistent with the angle change trajectory collected by the dynamic attitude analysis system. The angle trajectories of the hip and knee joints measured by the absolute angle sensor are the same as those obtained by the dynamic attitude analysis system. 1.5 rad and 0.3 rad were selected as reasonable and effective thresholds for determining sitting and standing states.

## 1. Introduction

In recent years, in the field of nervous system diseases, some progress has been made in the research on the rehabilitation of the central nervous system (CNS). Experts have found that the central nerves such as the brain and spinal cord can stimulate the nervous system of the lost limbs through repeated learning and training in a passive form, so that its function is restored and strengthened [1]. Therefore, an auxiliary system can be developed to drive the limbs to carry out repeated training and develop the potential learning function of the limbs. The higher the intelligent degree of the auxiliary system, the closer it is combined with the theory of human kinematics and the higher the success rate of lower limb rehabilitation [2, 3]. This restricts the implementation of the rehabilitation plan.

The research of rehabilitation robot field originates from the development and maturity of military exoskeleton industry. Industrial control technology and mechanical manufacturing technology have developed rapidly in the middle of last century. The research of the enhanced exoskeleton robot system started in the 1960s. In 1960, the United States General Electric Company developed the Hardiman series of exoskeleton robots, hoping to help the wearer lift a weight of up to 700 kg [4]. However, due to the restriction of objective factors such as industrial technology, the project goal was not fully achieved and only one arm was completed [2]. Although GE eventually stopped the project, Hardiman set the stage for enhanced exoskeletons, and the scientific community has continued to work on them. Today, there are a variety of enhanced exoskeletons that have been put into production.

With the rapid development of industrial technology, advanced science and technology are introduced into rehabilitation training, and a wearable rehabilitation robot system is formed by combining robotics, mechatronics, biological rehabilitation, intelligent control, information fusion, and rehabilitation medicine theories [5]. The rehabilitation robot system is mainly composed of four parts: the perception system, the control system, the mechanical mechanism (including the executive mechanism), and the power supply system. The perception system acquires the current motion mode, determines the wearer's motion intention, and provides a decision signal to the control system. The control system analyzes and determines the signal, forms the control signal, and assists the rehabilitation robot to complete the corresponding movement through the executive system. During this process, the perception system monitors the current motion mode in real time and the auxiliary control system controls.

Based on the research status of the rehabilitation robot perception system at home and abroad, combined with the characteristics of rehabilitation robot audience, the kinematics analysis system of human lower limbs was developed and designed, and on this basis, the sensing system of the wearable lower limb rehabilitation robot was studied.

The wearable health monitoring system is a typical application of wearable computing in the field of medicine. Wearable sensor-based monitoring of external vital signs in clinical settings ensures better support for assessing a patient's health status and can send automatic alerts to care providers in the event of health deterioration [6, 7]. Argent et al. evaluated a sample sensor-based biofeedback system and explored the feasibility, availability, perceived impact, and user experience of using the platform.

At present, the research on the monitoring system of wearable sensors is developing continuously. Jie et al. proposed a wearable human body monitoring system based on wireless acceleration sensor technology, which is used to real-time monitor the daily exercise amount of human body [8]. Ivacu et al. proposed different types of agents to process different sensor signals and identify simple daily life activities [9]. Chander et al. discussed wearable sensor networks for patient health monitoring: challenges, applications, future directions, and acoustic sensor challenges [10]. Zhou et al. proposed a wearable health monitoring system architecture based on human motion state recognition [11]. Simonetti et al. promoted the development of wearable tools and protocols to support functional rehabilitation of lower limb amputees by providing clinically relevant quantitative data [12]. Kshirsagar et al. proposed a wearable sensor network system for the safety and health application of the Internet of Things [13]. With exercise rehabilitation training as the background, Jiang et al. developed an exercise rehabilitation monitoring system based on wearable sensors and Internet of Things technology based on the Internet of Things technology [14]. Hung et al. applied the vulnerability index based on wearable sensors to the vulnerability classification of the elderly [15]. Gao et al. proposed a motion prediction model based on wearable sensors [16].

The main research is to design the perception system of the lower limb wearable rehabilitation robot, establish the kinematics theoretical model of the human lower limb, conduct the kinematics analysis of the human body, design the hardware circuit of the perception system, study the algorithm of the perception of the human body, and finally carry out the experimental verification on the industrial computer platform. The results show that the angle of the hip joint changes regularly between 0° and 37° and the angle of the knee joint changes regularly between 0° and 70° during the standing process, which is consistent with the angle change trajectory collected by the dynamic attitude analysis system. The angle trajectories of the hip and knee joints measured by the absolute angle sensor are the same as those obtained by the dynamic attitude analysis system. 1.5 rad and 0.3 rad were selected as reasonable and effective thresholds for determining sitting and standing states.

## 2. Research Methods

### 2.1. Sensor Layout

The motion feedback information selected by the perceptual system of a rehabilitation robot is as follows. Lower extremity EMG signal: collect and amplify muscle bioelectric information. EMG signal can be measured according to muscle activity before exercise, which can effectively make the rehabilitation robot and user move synchronously. However, EMG signals cannot be collected for patients with lower limb disability and loss of motor ability. Contact force information: collect and process the contact force between the rehabilitation robot parts and the ground force, as well as the contact force between the human and the rehabilitation equipment, and determine the current motion state and the movement intention of the user according to the size and distribution change of the force. Because the pressure sensor has some shortcomings such as nonlinearity, it needs to work with other sensor signals. Because there are too many contact points between human lower limbs and the rehabilitation robot system, it is impossible to determine and accurately place the contact force sensor to accurately locate the contact force [17]. Relatively speaking, the bottom of the foot pressure distribution is very regular, the pressure sensor can be placed in the heel of the foot, the second metatarsal, and the third metatarsal three places. Angle information: measure the instant angle of hip joint and knee joint to determine the current posture. Angular acceleration and linear acceleration information: the sensor is placed on the back, lower limbs, thighs, and calves to measure and analyze the angular acceleration and linear acceleration information of the sensor installation site to obtain the motion information of the current site.

In summary, the motion feedback signals that need to be collected in this project are determined as follows: plantar pressure information, joint angle information, angular acceleration information of back and lower limbs, and linear acceleration information.  Table 1 provides the type, quantity, and function of sensors [18]. The mechanical structure of the rehabilitation robot adds a crutch structure to help the wearer maintain balance and prevent falling. The angular acceleration sensor placed on the crutch can detect the swinging angle of the crutch and establish the current orientation of the crutch. A touchdown pressure switch is installed at the lower end of the crutch. The pressure switch has only two switch signals of 0 and 1. When the crutch touches the ground, the pressure switch is opened.

As shown in Figure 1, the sole pressure sensor should be placed at the heel of the sole, the second metatarsal bone, and the third metatarsal bone, and the pressure switch should be placed at the bottom of the crutches. The gyroscope/acceleration sensor is placed directly above the waist and on the upper side of the walking stick. The encoder is placed at the hip joint and knee joint.

### 2.2. Research on the Walking Process Perception Algorithm

When the wearer is in a standing posture, the movement intention is judged by the ground force distribution and the deviation of the center of gravity. The wearer extends the left crutch/right crutch forward, while the upper torso tilts to the left/right front, indicating that the wearer wishes to step forward with the right/left leg [19, 20]. Determine the movement intention from the angle of the torso. The movement intention of the patient can be obtained by measuring the acceleration angle signal (*θ*_*lg*_, *θ*_*rg*_) of the crutch and the direction of the pressure switch (*f*_*lg*_, *f*_*rg*_) of the crutch bottom.

(1) $$\begin{array}{c} \theta_{lg}>\theta_{+}, \end{array}$$

(2) $$\begin{array}{c} \theta_{rg}<\theta_{-}, \end{array}$$

(3) $$\begin{array}{c} f_{\mathrm{lg}}=ON, \end{array}$$

(4) $$\begin{array}{c} f_{rg}=ON. \end{array}$$

Walking intention is divided into swinging the right leg and swinging the left leg. When (1) and (3) are satisfied, the rehabilitation robot assists to take the right leg; when (2) and (4) are satisfied, the rehabilitation robot assists to take the left leg. In the process of walking, if the heel pressure *f*_*lh*_ or *f*_*rh*_ of the swinging leg is greater than the threshold value *f*_*s*_, the leg support phase is entered. If the swing of the walking stick stops and the swing of the trunk stops at the same time, the wearer is considered to have the intention to stop walking, and the rehabilitation robot will assist in walking and change to a standing state.

In the process of rise, sit, and walk through the foot pressure acquisition of real-time detection of horizontal axis ZMP information, if the ZMP stable signal exceeds the threshold (one foot in the threshold size of rehabilitation robots length), namely, the rehabilitation robot system is in unstable condition, need to issue instructions to the control system, make its provide auxiliary torque, and restores the balance of the healing machine. Equation (5) should be satisfied for the rehabilitation robot to maintain balance:

(5) $$\begin{array}{c} x_{zmp}\leq la, \end{array}$$

where *l*_*a*_ is the length of the rehabilitation robot's single foot.

### 2.3. IPC-Based Experimental Verification Platform

IPC has the characteristics of easy transplantation and powerful computing power. The development and verification platform of experimental methods and algorithms can be built on IPC, which can greatly shorten the development cycle. At the same time, the data acquisition card can be used to analyze the collected signals conveniently, which provides a basis for algorithm research.

IPC experimental verification platform refers to the hardware system of IPC and the supporting software based on this hardware. In the rehabilitation robot system, the IPC experimental verification platform includes PC, signal acquisition board card, sensor signal acquisition module, Matlab software and Visual Studio software.

A software debugging platform based on Matlab + Simulink and ADAMS software is developed based on IPC hardware platform. ADAMS is a software for the analysis of kinematics, dynamics, and statics of mechanical structures developed by MDI Corporation (now incorporated into MSC Software Corporation) in America. The body limb model was established by ADAMS, and the mechanical structure of the rehabilitation robot system was simulated and optimized. The moment of inertia of each limb is calculated to provide reference data for the selection of the actuator.

During the experiment, after wearing the rehabilitation robot, the posture was first adjusted to the sitting or standing state, and after the judgment was completed, the corresponding state transition actions were made to express the motion intention, namely, the intention of standing while sitting and the intention of standing or walking while standing. After the rehabilitation robot assists to complete the corresponding action, it makes the next state transition action again. The rehabilitation robot can detect the current posture and judge the movement intention to carry out the next auxiliary action.

## 3. Results Analysis and Discussion

Through D/A transformation, filtering, and other processing, the PIC microcontroller transmits the foot pressure to the top computer through CAN bus and obtains the real-time pressure information through the digital filtering circuit.

First, the FlexiForce thin film pressure sensor is calibrated. Place the nominal weight on the FlexiForce sensor, record the voltage values, and draw a table as given in Table 2. The pressure range is 0–500 N, each test increases by 50 N, and the output voltage is converted to 0–5 V through AD.

The pressure-voltage curve is drawn as shown in Figure 2. It can be seen that the FlexiForce sensor has good linear correlation. When the pressure varies from 0 to 500 N, the voltage value is output linearly from 0 to 5 V. The relationship between foot pressure and voltage reading can be obtained by fitting:

(6) $$\begin{array}{c} \frac{F}{V}=100. \end{array}$$

The detection and drawing of the pressure distribution of six foot pressure sensors in different motion states are carried out. After filtering, the foot pressure distribution map can be obtained in the walking process and the standing process.

Combined with phase differentiation, the pressure distribution of feet in a gait cycle is analyzed, as shown in Figure 3. The horizontal axis is time in seconds, and the vertical axis is pressure in cattle. The solid line is the pressure distribution of the heel, the dotted line is the pressure distribution of the second phalangeal bone on the sole of the foot, and the dotted line is the pressure distribution of the fifth phalangeal bone on the sole of the foot. In the process of walking, the foot pressure showed regular changes, appeared in the process of walking foot toe bone in 2 foot pressure peaks value, peak about 320 N, the foot phalanges place 5 foot pressure peaks appeared before the second toe bone, peak at about 150 N, and the heel stress peak reached before a toe pressure peak value, the peak is around 100 N.

As can be seen from Figure 4, in the process of walking, the sole pressure of the foot presents regular distribution in each walking cycle. When entering the leg support phase, the pressure on the heel begins to increase and the pressure on the second metatarsal is at a high value. When entering the single-leg swing phase, the pressure on the supporting foot becomes excessive from the heel to the sole of the foot. The method of the threshold value is used to determine the current state of motion and predict the trend of motion.

GOF information of lower limbs can be detected through the information of foot pressure. The switching rules of GOF information during walking are as follows: the left leg enters the swing phase, the right leg starts in the support phase, and the left leg swings to the highest point. In the horizontal plane, the GOF changes from left back to right front. When the left leg swings to the highest point and the left foot falls to the ground completely, the right leg enters the swing phase. During this process, the change of GOF in the horizontal plane changes from right back to left front. When moving forward, the right leg of the lower limb enters the swing phase and swings to the highest point of the right leg. In the horizontal plane, GOF changes from right back to left front. The right leg starts to swing to the highest point until the right foot completely lands, and the left leg enters the swing phase. During this process, the GOF changes from left back to right front in the horizontal plane. At this point, a periodic gait process is completed, during which the trajectory of GOF also completes a periodic change. In one cycle, the change in the horizontal plane is left back to right front, right back to left front, and left back to right front.

The angle of hip joint and knee joint measured by the OMRON absolute angle encoder was transmitted to the top computer, and the absolute angle changes of hip joint and knee joint were obtained during the process of standing up, sitting up, and walking. In the process of standing up, when the angular velocity of the knee joint reaches the maximum value, the time point is about 70% of the whole standing up process, so it is reasonable and effective to select this point as the phase conversion point in the standing up process.

The angle trajectories of the hip and knee joints measured by the absolute angle sensor are the same as those obtained by the dynamic attitude analysis system. 1.5 rad and 0.3 rad were selected as reasonable and effective thresholds for determining sitting and standing states.

## 4. Conclusions

The lower limb motion state transition model based on a finite state machine was established, the human body sensing algorithm was studied, the sensor group information was collected and fused, the current motion mode was judged, and the algorithm to determine the human motion intention was verified. The signal of the sensor group enters the signal acquisition board for centralized preprocessing, and then, it is sent to the industrial computer. The industrial computer calculates the sensor signal, locates the current motion mode of the wearer, and perceives the motion intention of the wearer through the perception algorithm. With the rapid development of industrial technology, advanced science and technology introduced rehabilitation training, using the combination of robotics, electromechanical technology, biological rehabilitation technology, intelligent control technology, information integration technology, rehabilitation medicine, form a wearable rehabilitation robot system, created the first of enhanced exoskeleton research, and research institutions in the field of enhanced exoskeleton. By comparing the experimental results with the theoretical results of the perceptual algorithm, the perceptual algorithm is verified. The experimental results show that the angle of the hip joint changes regularly between 0° and 37° and that of the knee joint changes regularly between 0° and 70°, which is consistent with the trajectory of angle change collected by the dynamic attitude analysis system. The angle trajectories of the hip and knee joints measured by the absolute angle sensor are the same as those obtained by the dynamic attitude analysis system. 1.5 rad and 0.3 rad were selected as reasonable and effective thresholds for determining sitting and standing states.

## Figures and Tables

**Figure 1:** Distribution diagram of sensor selection.

**Figure 2:** Pressure and voltage corresponding diagram.

**Figure 3:** Pressure distribution of feet during walking.

**Figure 4:** Foot pressure distribution in a gait cycle.

**Table 1:** Sensor selection of the perception system.

The sensor	Installation position	Measure the signal	Use
Pressure sensor, pressure switch	A pressure switch is placed on the bottom of the crutch, and 3 pressure sensors are placed on each sole	The reaction of the earth to the wearer	The gait of the wearer is judged as feedback information for the correction and control of gait prediction

Gyroscope/acceleration sensor	Lower back, upper part of crutches (3)	Angular acceleration and linear acceleration	Obact, the movement state of the body and the walking stick and judge the walking intention of the wearer

The encoder	Hip joint, knee joint (4)	Joint angle	Determine the current motion mode

**Table 2:** FlexiForce pressure calibration values.

Pressure (N)	0	25	50	75	100	125	150	175	200

Voltage (V)	0	0.23	0.52	0.77	1.04	1.24	1.52	1.73	2.03
Pressure (N)	225	250	275	300	325	350	375	400	425
Voltage (V)	2.4	2.45	2.77	3.04	3.24	3.55	3.73	3.96	4.23
Pressure (N)	450	475	500						
Voltage (V)	4.46	4.72	4.95						

## Data Availability

The data used to support the findings of this study are available from the corresponding author upon request.

## References

[1] Zhang S.-H., Wang F.-X., Li J.-J., Peng H.-D., Yan J.-H., Pan G.-B. (2017). Wearable wide-range strain sensors based on ionic liquids and monitoring of human activities. *Sensors*.

[2] Ritika, Ramachandran A. (2019). Wearable sensors: a step towards smart monitoring of high risk pregnancies. *International Journal of Scientific & Technology Research*.

[3] Ma B., Nie S., Ji M., Song J., Wang W. (2020). Research and analysis of sports training real-time monitoring system based on mobile artificial intelligence terminal. *Wireless Communications and Mobile Computing*.

[4] Cao W.-J., Hu J., Wang Z.-P., Wang L.-L., Yu H.-L. (2017). Study on a novel wearable exoskeleton hand function training system based on emg triggering. *Wearable Sensors and Robots*.

[5] Bloss R. (2015). Wearable sensors bring new benefits to continuous medical monitoring, real time physical activity assessment, baby monitoring and industrial applications. *Sensor Review*.

[6] Rodriguez V. H., Medrano C. T., Plaza I. (2018). Wearable sensors for measuring movement in short sessions of mindfulness sitting meditation: a pilot study. *Journal of Healthcare Engineering*.

[7] Bobić V., Djurić-Jovičić M., Dragašević N., Popović M. B., Kostić V. S., Kvaščev G. (2019). An expert system for quantification of bradykinesia based on wearable inertial sensors. *Sensors*.

[8] Jiang P., Winkley J., Zhao C., Munnoch R., Min G., Yang L. T. (2016). An intelligent information forwarder for healthcare big data systems with distributed wearable sensors. *IEEE Systems Journal*.

[9] Ren J., Guan F., Pang M., Li S. (2020). Monitoring of human body running training with wireless sensor based wearable devices. *Computer Communications*.

[10] Ivașcu T., Negru V. (2021). Activity-Aware Vital Sign Monitoring Based on a Multi-Agent Architecture. *Sensors*.

[11] Chander B., Kumaravelan (2021). Wearable sensor networks for patient health monitoring: challenges, applications, future directions, and acoustic sensor challenges. *Healthcare Paradigms in the Internet of Things Ecosystem*.

[12] Zhou X. (2020). Wearable health monitoring system based on human motion state recognition. *Computer Communications*.

[13] Conradsson D., Nero H., Lfgren N., Hagstrmer M., Franzén E. (2017). Monitoring training activity during gait-related balance exercise in individuals with Parkinson’s disease: a proof-of-concept-study. *BMC Neurology*.

[14] Kshirsagar P. (2021). A wearable sensor network system for iot-connected safety and health applications. *Journal of Information Storage and Processing Systems*.

[15] Tonacci A., Dellabate A., Dieni A. (2020). Can machine learning predict stress reduction based on wearable sensors’ data following relaxation at workplace? a pilot study. *Processes*.

[16] Boissy P., Blamoutier M., Brière S., Duval C. (2018). Quantification of free-living community mobility in healthy older adults using wearable sensors. *Frontiers in Public Health*.

[17] Gao T., Lou Y., Sivaparthipan C. B., Alazab M. (2021). Prediction of athlete movements using wearable sensors for sports person health monitoring application. *Journal of Intelligent & Fuzzy Systems*.

[18] Hui P. (2018). Stretchable health sensor could improve monitoring of chronic conditions. *Fiber Optic Sensors and Systems*.

[19] Zhang K., Ling W. (2020). Health monitoring of human multiple physiological parameters based on wireless remote medical system. *IEEE Access*.

[20] Berthelot M., Henry F. P., Hunter J., Leff D., Wood S., J Allali N. (2019). Pervasive wearable device for free tissue transfer monitoring based on advanced data analysis: clinical study report. *Journal of Biomedical Optics*.

